The article "Zonisamide's Efficacy and Safety on Parkinson's Disease and Dementia with Lewy Bodies: A Meta-Analysis and Systematic Review" was retracted in 2024. Reasons: signs of a paper mill; suspected computer-generated content; unreliable results or conclusions; lack of ethics approval or compliance.

# Zonisamide's Efficacy and Safety on Parkinson's Disease and Dementia with Lewy Bodies: A Meta-Analysis and Systematic Review

**DOI:** 10.1155/2022/4817488

**Published:** 2022-09-12

**Authors:** Linghui Kong, Jiaqiu Xi, Zhenyuan Jiang, Xiaowen Yu, Hailiang Liu, Zhonglin Wang

**Affiliations:** ^1^The First Clinical Medical College, Shandong University of Chinese Medicine, Jinan, China; ^2^Shandong Hospital of Traditional Chinese Medicine, Jinan, China

## Abstract

**Objective:**

Clinical data has recently shown an association between Parkinson's disease (PD), Dementia with Lewy bodies (DLB), and zonisamide. The purpose of this study was to thoroughly evaluate the efficacy and safety of zonisamide in PD and DLB.

**Methods:**

Pubmed, the Cochrane Library, Web of Science, and Embase databases were searched for all randomized clinical trials (RCTS) on the role of zonisamide in PD and DLB that were completed by April 18, 2022. UPDRS II (off) total score, UPDRS III total score, Daily “off” time, and UPDRS Part IV, Nos. 32, 33, and 34 were used as clinical efficacy endpoints. Adverse events reported in the RCTs will be considered in the final safety analysis. To better understand the effect of zonisamide on the efficacy and safety of PD and DLB, the UPDRS III total score and the six overlapping adverse events were examined in subgroups. Either a fixed effects model analysis (OR) or a random effects model analysis (MD) is used to figure out the mean difference (MD) and the relative risk.

**Results:**

Seven articles involving 1749 patients (916 PD and 833 DLB) were included in this study. Compared to the control group, zonisamide could significantly reduce the UPDRS III total score in patients with PD and DLB (WMD-2.27 [95% CI: -3.06, -1.48], *p* < 0.0001). For patients with PD, compared to the control group, zonisamide could significantly reduce the UPDRS II (off) total score (WMD-0.81 [95% CI: -1.36, -0.26], *p* = 0.004), daily “off” time (WMD-0.67 [95% CI: -1.10, 0.24], *p* = 0.002), and UPDRS part IV, No. 32 worsen (OR-3.48 [95% CI: 1.20, 10.10], *p* = 0.02). In terms of safety, compared with the control group, for patients with DLB, zonisamide could significantly increase the incidence of contusion (OR-0.60 [95% CI: 0.38, 0.96], *p* = 0.03) and may increase the probability of reduced appetite (OR-3.13 [95% CI: 1.61, 6.08], *p* = 0.0008). And for patients with PD, zonisamide may increase the probability of somnolence (OR-2.17 [95% CI: 1.25, 3.76], *p* = 0.006).

**Conclusions:**

For the analysis of the current study results, our results show that zonisamide could improve the motor function in patients with PD and DLB and improve the activities of daily living (off) and wearing off and decrease the duration of dyskinesia in patients with PD. In terms of safety, the use of zonisamide significantly increases the probability of contusion in patients with DLB and may increase the probability of reduced appetite in patients with DLB and somnolence in patients with PD. Zonisamide appears to be a new treatment option for patients with PD and DLB. However, the effectiveness and safety of zonisamide in the treatment of PD and DLB need to be further investigated.

## 1. Introduction

Parkinson's disease (PD) is the second most common neurodegenerative disease, with a prevalence of 0.3-1.0% in the general population and about 1-3% in people aged > 60 years [1–3]. The core feature of clinical PD is motor syndrome, defined as bradykinesia, in combination with either rest tremor, rigidity, or both [4]. Due to the growing population's aging, both the prevalence and incidence of PD are expected to rise by at least 30% by 2030, which will place additional strain on society and the global economy [5]. Dementia with Lewy bodies (DLB) is the second most common form of dementia after Alzheimer's disease, accounting for 10–20% of all dementia cases [6, 7]. The central feature of DLB is progressive cognitive decline, with core clinical features including fluctuating cognition, recurrent visual hallucinations, rapid eye movement, sleep behavior disorder, and parkinsonism. DLB and PD belong to the same spectrum of diseases and have similar pathology, mainly in the form of a large number of alpha-synuclein-based Lewy bodies in the brain and autonomic nervous system [8, 9]. In the clinical management of PD and DLB, levodopa has been mentioned repeatedly and is particularly critical.

For PD patients, dopamine replacement therapy is currently the primary method of improving motor symptoms in Parkinson's disease, and while it helps to improve motor performance temporarily, it does not help to slow down the neurodegenerative process. In addition, the prolonged use of levodopa can lead to motor complications, including hypokinesia and dyskinesia [10], which can have severe effects on activities of daily living and quality of life [11–13]. Therefore, the improvement of wearing off without the worsening of dyskinesia is a therapeutic goal in patients with PD who experience wearing off [14], whereas for DLB patients, they usually respond less to dopaminergic treatment than PD patients. Even though some DLB patients may benefit from levodopa preparations to improve their own dyskinesia, the doses used are severely limited and do not achieve the best improvement due to concerns about worsening neuropsychiatric symptoms, including delirium and BPSD [15, 16]. Therefore, the improvement of levodopa in both PD and DLB patients is relatively limited and does not last consistently for a long period of time.

Zonisamide (1,2-benzisoxazole-3-methanesulfonamide) was discovered in Japan in 1974 as a sulphonamide with anticonvulsant properties and is widely used clinically for the treatment of partial-onset epilepsy and mixed epilepsy [17]. Zonisamide's pharmacological profile is complicated, and it has a lot of binding targets. The pharmacological mechanisms that have been confirmed so far are mainly inhibitory activities on voltage-gated sodium channels, T-type calcium channels, and MAO-B [18]. In addition, it has also been shown to have neuromodulatory effects on a variety of neurotransmitter systems, including cholinergic, serotonergic, glutamatergic, and monoaminergic systems in clinical trials [19]. The potential beneficial effects of zonisamide in relation to the nervous system have been progressively demonstrated in a variety of neurological disorders, including migraine, PD, neuropathic pain, and mood disorders [20, 21].

Initially, zonisamide showed an unexpected improvement in dyskinesia in the clinical treatment of epilepsy patients in combination with PD. Numerous clinical trials, case series, observational studies, and case reports have been published since then to support the efficacy of zonisamide in PD and DLB. Therefore, zonisamide could be a promising drug candidate for the treatment of PD and DLB. There is no comprehensive analysis of RCTs of zonisamide in PD and DLB; so, we conducted this study to investigate the efficacy and safety of zonisamide in PD and DLB.

## 2. Methods

### 2.1. Data Sources and Search Strategy

The design of this study was based on the results of a systematic review and meta-analysis (PRISMA) [22]. The protocol for this study was registered with PROSPERO [23]. We used the following databases to conduct an electronic search: Pubmed, Cochrane library, Web of science, and Embase are all available online. The following were the subject terms: “PD,” “DLB,” and “zonisamide.” There are no restrictions on language, and the most recent search was conducted on April 18,2022.

### 2.2. Selection and Eligibility Criteria

Two reviewers independently screened the search results for titles, abstracts, and full text reviews, and disagreements were settled through consensus or discussion with a third independent author. RCTs on the efficacy of zonisamide in the treatment of PD and DLB are among the inclusion criteria. There were only original articles included. The following were the exclusion criteria: non-RCTs, nonhuman studies, duplicates, conference papers, meta-analyses, or systematic reviews.

### 2.3. Data Extraction and Outcomes

The reviewers extracted relevant data from each study independently into predesigned Excel spreadsheets, which included the following: country of origin; year of publication; and the first author; study duration; study population; intervention; number, sex, and age of participants; comorbidities; duration of PD or DLB; baseline patient data; and treatment outcomes. Among the outcomes were the UP-DRS II (activities of daily life) total score, the UPDRS III (motor function) total score, and the daily “off” time. UPDRS Part IV, No. 32 (duration of dyskinesia) includes the following: worsened, improved, no new onset, unchanged with scores ≥ 1, and new onset. UPDRS Part IV, No. 33 (disability caused by dyskinesia) includes the following: worsened, improved, no new onset, and unchanged with scores ≥ 1. UP-DRS Part IV, No. 34 (pain caused by dyskinesia) includes the following: worsened, improved, no new onset, and unchanged with scores ≥ 1. In addition, 39 adverse events were included as indicators of treatment safety outcomes. We calculated the means and standard deviations for continuous dating (MD). The data were transformed using existing formulae in the absence of a mean and standard deviation. A third reviewer resolved disagreements independently.

### 2.4. Statistical Analysis and Quality Assessment

Statistical analysis was performed using Review Manager 5.4. We analyzed continuous variables using standardized mean differences (SMD) and 95% confidence intervals (CI). The *I*^2^ statistic was used to evaluate heterogeneity. *I*^2^ values of 25%, 50%, and 75% were considered low, medium, and high heterogeneity, respectively. To summarize the data from all studies, random-effects models were used. Statistical significance was defined as *P* values less than 0.05. The funnel plot will be used to assess the risk of publication bias in studies. The Cochrane Risk of Bias Assessment Tool was used to evaluate the RCT's quality, which included six criteria: randomized sequence generation, allocation concealment, patient blindness, trial participants, outcome evaluator blindness, incomplete outcome data, selective reporting, and other biases.

## 3. Results

### 3.1. Search Results

673 studies were identified through the literature search, 112 of which were from PubMed, 60 from the Cochrane Library, 134 from the Web of Science, and 367 from Embase. After excluding 229 duplicates and reviewing 444 titles and abstracts, 435 outcomes were excluded, and the remaining 9 outcomes were reviewed in detail. A total of 7 RCTs were included in the meta-analysis, of which three RCTs were conducted on patients with DLB, and the other four RCTs were conducted on patients with PD [24–30]. The study selection process is summarized in the PRISMA flow chart in Figure 1.

### 3.2. Study Characteristics and Quality Assessment

Seven studies were conducted between 2007 and 2021, with a total of 1749 additional participants (in the experimental group, 1181 participants used zonisamide, while in the control group, 569 participants used a placebo). All patients were diagnosed with PD or DLB (all patients were asked to use concomitant levodopa preparations (including DCI combination drugs), and patients can continue to use other anti-Parkinson drugs such as dopamine agonists (DA), monoamine oxidase type B (MAO-B) inhibitors, amantadine or droxodopa, and anticholinergics during the study period. For patients with DLB, they were also allowed to continue using antidementia drugs during the study (specific drug type not mentioned). These concomitant doses and dosing regimens should remain stable for at least 4 weeks prior to the start of the formal study until the end of the study, and patients who are unable to follow these principles are considered to have dropped out of the final analysis. All of the studies were conducted in Japan, and the interventions lasted anywhere from 14 to 52 weeks, with the exception of the first RCTs (the earliest study), and the exclusion criteria were set for the remaining six RCTs to ensure that there was no overlap of patients in the study. According to the Cochrane Risk of Bias tool, seven RCTs were parallel-group studies and articles of generally moderate and high quality. The results of the seven RCTs' quality evaluations are summarized in Figures 2(a) and 2(b).

### 3.3. The Effect of Zonisamide on UPDRS III Total Score

A total of 7 RCTs reported the UPDRS III total score in 1636 patients (1094 zonisamide users and 542 nonusers). Four RCT studies included PD patients, and the other three included DLB patients. Our analysis demonstrated that zonisamide obviously reduces the UPDRS III total score among all patients compared with controls, which had statistical differences (WMD-2.27 [95% CI: -3.06,-1.48], *p* < 0.00001). There was low heterogeneity between studies (*p* = 0.04, *I*^2^ = 45%) (Figure 3(a)). In addition, our subgroup analysis showed that zonisamide significantly reduced the UPDRS III total score for both PD patients and DLB patients. And the results were all statistically significant (PD: (WMD-1.83 [95% CI: -2.53, -1.13], *p* < 0.00001) DLB: (WMD-2.09 [95% CI: -2.64, -1.53], *p* < 0.00001) (Figure 3(b)). By comparing subgroup differences, the effect of zonisamide in reducing the UPDRS III total score appears to be more pronounced in patients with DLB.

### 3.4. The Effect of Zonisamide on UPDRS II “Off” Total Score

A total of 3 RCTs reported the UPDRS II “off” total score in 538 PD patients (348 zonisamide users and 190 nonusers). The meta-analysis concluded that zonisamide reduced the UPDRS II “off” total score in PD patients compared to controls. There was a significant statistical difference (WMD-0.81 [95% CI: -1.36,-0.26], *p* = 0.004). There was low heterogeneity between studies (*p* = 0.33, *I*^2^ = 13%) (Figure 3(c)).

### 3.5. The Effect of Zonisamide on Daily “Off” Time

A total of 2 RCTs reported the daily “off” time of 614 patients (424 zonisamide users and 190 nonusers). Our study found that zonisamide significantly reduces daily “off” time in PD patients when compared to controls with statistically significant differences (WMD-0.67 [95% CI: -1.10, 0.24], *p* = 0.002). There was moderate heterogeneity between studies (*p* = 0.05, *I*^2^ = 57%), and through intragroup subgroup analysis, we observed that medium heterogeneity may be due to dose difference. (Figures 3(d) and 3(e)).

### 3.6. The Effect of Zonisamide on UPDRS IV, No. 32

#### 3.6.1. Worsened

A total of 2 RCTs reported the UPDRS IV, No. 32 worsened in 285 patients (194 zonisamine users and 91 nonusers). Our study found that zonisamide significantly reduces the UPDRS IV No. 32 worsened in PD patients when compared to controls, with statistically significant differences (OR-3.48 [95% CI: 1.20, 10.10], *p* = 0.02). There was no evidence of heterogeneity between studies (*p* = 0.88, *I*^2^ = 0%) (Figure 4(a)).

#### 3.6.2. Improved

A total of 2 RCTs reported the UPDRS IV, No. 32 improved in 285 patients (194 zonisamide users and 91 nonusers). When compared to controls, zonisamide was likely to increase the UPDRS IV, No. 32 improved in patients with PD. However, statistical diversity was limited (OR-0.92 [95% CI: 0.34, 2.55], *p* = 0.88). There was low heterogeneity between studies (*p* = 0.28, *I*^2^ = 22%) (Figure 4(b)).

#### 3.6.3. No New Onset

A total of 1 RCTs reported UPDRS IV, No. 32 no new onset in 185 patients (122 zonisamide users and 63 nonusers). When compared to controls, zonisamide was likely to reduce the UPDRS IV, No. 32 no new onset in patients with PD. However, statistical diversity was limited (OR-0.92 [95% CI: 0.49, 1.72], *p* = 0.79). There was low heterogeneity between studies (*p* = 0.29, *I*^2^ = 10%) (Figure 4(c)).

#### 3.6.4. Unchanged with Scores ≥ 1

A total of one RCTs reported UPDRS, IV No. 32 unchanged with scores ≥ 1 in 185 patients (122 zonisamine users and 63 nonusers). When compared to controls, zonisamide was likely to increase the UPDRS, IV No. 32 unchanged with scores ≥ 1 in patients with PD. However, statistical diversity was limited (OR-0.98 [95% CI: 0.51, 1.90], *p* = 0.96). There was no evidence of heterogeneity between studies (*p* = 0.61, *I*^2^ = 0%) (Figure 4(d)).

#### 3.6.5. New Onset

A total of 1 RCTs reported UPDRS IV, No. 32 new onset in 185 patients (122 zonisamide users and 63 nonusers). When compared to controls, zonisamide was likely to increase the UPDRS IV, No. 32 new onset in patients with PD. However, statistical diversity was limited (OR-4.16 [95% CI: 0.45, 38.14], *p* = 0.21). There was no evidence of heterogeneity between studies (*p* = 0.82, *I*^2^ = 0%) (Figure 4(e)).

### 3.7. The Effect of Zonisamide on UPDRS IV, No. 33

#### 3.7.1. Worsened

A total of 2 RCTs reported the UPDRS IV, No. 33 worsened in 424 patients (278 zonisamine users and 146 nonusers). The effect of zonisamine on UPDRS IV, No. 33 worsened was not statistically significant when compared to the control group (OR-0.50 [95% CI: 0.21, 1.20], *p* = 0.12). There was no evidence of heterogeneity between studies (*p* = 0.43, *I*^2^ = 0%) (Figure 5(a)).

#### 3.7.2. Improved

A total of 2 RCTs reported the UPDRS IV, No. 33 improved in 424 patients (278 zonisamine users and 146 nonusers). The effect of zonisamine on UPDRS IV, No. 33 improved was not statistically significant when compared to the control group (OR-1.60 [95% CI: 0.78, 3.28], *p* = 0.2). There was no evidence of heterogeneity between studies (Figure 5(b)).

#### 3.7.3. Unchanged with Scores ≥ 1

A total of one RCTs reported the UPDRS IV, No. 33 unchanged with scores ≥ 1 in 375 patients (246 zonisamide users and 129 nonusers). The effect of zonisamine on UPDRS IV, No. 33 unchanged with scores ≥ 1 was not statistically significant when compared to the control group (OR-0.75 [95% CI: 0.38, 1.46], *p* = 0.4). There was no evidence of heterogeneity between studies (*p* = 0.66, *I*^2^ = 0%) (Figure 5(c)).

#### 3.7.4. Zero (No New Onset)

A total of 1 RCTs reported the UPDRS IV, No. 33 zero in 375 patients (246 zonisamine users and 129 nonusers). The effect of zonisamine on UPDRS IV, No. 33 zero was not statistically significant when compared to the control group (OR-1.14 [95% CI: 0.70, 1.88], *p* = 0.59). There was no evidence of heterogeneity between studies (*p* = 0.64, *I*^2^ = 0%) (Figure 5(d)).

### 3.8. The Effect of Zonisamide on UPDRS IV, No. 34

#### 3.8.1. Worsened

A total of 1 RCTs reported the UPDRS IV, No. 34 worsened in 375 patients (246 zonisamide users and 129 nonusers). The effect of zonisamine on UPDRS IV, No. 34 worsened was not statistically significant when compared to the control group (OR-0.73 [95% CI: 0.19, 2.72], *p* = 0.63). There was no evidence of heterogeneity between studies (*p* = 0.42, *I*^2^ = 0%) (Figure 6(a)).

#### 3.8.2. Improved

A total of 1 RCTs reported the No. 34 improved in 375 patients (246 zonisamide users and 129 nonusers). The effect of zonisamine on UPDRS IV, No. 34 improved was not statistically significant when compared to the control group (OR-1.57 [95% CI: 0.25, 9.72], *p* = 0.63). There was no evidence of heterogeneity between studies (*p* = 0.70, *I*^2^ = 0%) (Figure 6(b)).

#### 3.8.3. Unchanged with Scores ≥ 1

A total of one RCTs reported the UPDRS IV, No. 34 unchanged with scores ≥ 1 in 375 patients (246 zonisamide users and 129 nonusers). The effect of zonisamine on UPDRS IV, No. 34 unchanged with scores ≥ 1 was not statistically significant when compared to the control group (OR-2.05 [95% CI: 0.35, 11.96], *p* = 0.42). There was no evidence of heterogeneity between studies (*p* = 0.53, *I*^2^ = 0%) (Figure 6(c)).

#### 3.8.4. Zero (No New Onset)

A total of 1 RCTs reported the UPDRS IV, No. 34 zero in 375 patients (246 zonisamine users and 129 nonusers). The effect of zonisamine on UPDRS IV, No.34 zero was not statistically significant when compared to the control group (OR-0.88 [95% CI: 0.32, 2.43], *p* = 0.80). There was no evidence of heterogeneity between studies (*p* = 0.26, *I*^2^ = 0%) (Figure 6(d)).

#### 3.8.5. Adverse Events

Seven RCTs reported the results of a total of 39 adverse events. Six adverse events, including excoriation, rash, restless legs syndrome, hypnagogic hallucination, abnormal behavior, and attention deficit, were not included in the analysis due to incomplete data. A total of 33 adverse events were included in the analysis. In addition, we also performed subgroup analysis for six of them (contusion, somnolence, reduced appetite, constipation, weight loss, and insomnia) because they have been reported in RCTs of both PD and DLB with zonisamide.

## 4. Contusion

A total of 5 RCTs reported adverse events of contusion loss in 1421 patients (1048 zonisamide users and 373 nonusers) during the trial. Our analysis results showed that compared with the control group, zonisamide significantly increased the occurrence probability of contusion. There was a significant statistical difference (OR-0.59 [95% CI: 0.39, 0.89], *p* = 0.01). There was no significant difference in heterogeneity among included studies (*p* = 0.91, *I*^2^ = 0%) (Figure 7(a)). In addition, further subgroup analysis showed that for DLB patients, compared with the control group, zonisamide also significantly increased the occurrence probability of contusion. The results showed a statistical difference (OR-0.60 [95% CI: 0.38, 0.96], *p* = 0.03). However, for PD patients, there was no statistical difference between the placebo and zonisamide groups (OR-0.45 [95% CI: 0.19, 1.07], *p* = 0.07) (Figure 7(b)).

### 4.1. Somnolence

A total of 1592 RCTs (1078 zonisamide users and 514 nonusers) reported somnolence adverse events during the trial, and there was no significant difference in somnolence occurrence probability between the zonisamide group and the control group (OR-1.54 [95% CI: 0.96, 2.49], *p* = 0.07). There was low heterogeneity among included studies (*p* = 0.33, *I*^2^ = 12%) (Figure 7(c)). In addition, further subgroup analysis showed that for DLB patients, there was also no statistical difference between the placebo and zonisamide groups (OR-1.08 [95% CI: 0.58, 2.01], *p* = 0.81). However, for PD patients, compared with the control group, the results showed a statistical difference (OR-2.17 [95% CI: 1.25, 3.76], *p* = 0.006) (Figure 7(d)).

### 4.2. Reduced Appetite

A total of 1751 RCTs (1189 zonisamide users and 562 nonusers) reported reduced appetite and adverse reactions during the trial. There was no significant difference in the incidence probability of reduced appetite between the zonisamide group and the control group (OR-1.16 [95% CI: 0.68, 1.99], *p* = 0.58). There was low heterogeneity among the included studies (*p* = 0.06, *I*^2^ = 41%) (Figure 8(a)) In addition, further subgroup analysis showed that for PD patients, there was also no statistical difference between the placebo and zonisamide groups (OR-0.67 [95% CI: 0.43, 1.05], *p* = 0.08). However, for DLB patients, compared with the control group, the results showed a statistical difference (OR-3.13 [95% CI: 1.61, 6.08], *p* = 0.0008) (Figure 8(b)).

### 4.3. Weight Loss

A total of 4 RCTs reported adverse events of weight loss in 1012 patients (702 zonisamide users and 310 nonusers) during the trial, and there was no significant difference in the probability of weight loss between the zonisamide group and the control group (OR-1.29 [95% CI: 0.80, 2.09], *p* = 0.29). There was no significant difference in heterogeneity among included studies (*p* = 0.53, *I*^2^ = 0%) (Figure 8(c)). Further subgroup analysis also showed that there was no statistically significant difference in the incidence of weight loss between the zonisamide group and the control group for both PD and DLB patients (PD: (OR-1.01 [95% CI: 0.54, 1.89], *p* = 0.98) DLB: (OR-2.01 [95% CI: 0.85, 4.80], *p* = 0.11) (Figure 8(d)).

### 4.4. Constipation

A total of 5 RCTs reported 1593 patients (1089 zonisamide users and 504 nonusers) with bouts of constipation during the trial. There was no significant difference in the incidence rate of constipation between the zonisamide group and the control group (OR-0.95 [95% CI: 0.60, 1.53], *p* = 0.85). There was low heterogeneity among included studies (*p* = 0.43, *I*^2^ = 2%) (Figure 9(a)). Further subgroup analysis also showed that there was no statistically significant difference in the incidence of constipation between the zonisamide group and the control group for both PD and DLB patients (PD: (OR-1.16 [95% CI: 0.64, 2.10], *p* = 0.63), DLB: (OR-0.64 [95% CI: 0.34, 1.22], *p* = 0.18)) (Figure 9(b)).

### 4.5. Insomnia

A total of four RCTs reported 1263 patients (842 zonisamide users and 421 nonusers) with adverse insomnia during the trial, and there was no significant difference in the probability of insomnia between the zonisamide group and the control group (OR-0.78 [95% CI: 0.43, 1.43], *p* = 0.42). There was no significant difference in heterogeneity among included studies (*p* = 0.82, *I*^2^ = 0%) (Figure 9(c)). Further subgroup analysis also showed that there was no statistically significant difference in the incidence of insomnia between the zonisamide group and the control group for both PD and DLB patients (PD: OR-0.56 [95% CI: 0.26, 1.21], *p* = 0.14), DLB: OR-1.45 [95% CI: 0.51, 4.12], *p* = 0.49) (Figure 9(d)).

In addition, we performed a statistical analysis of the remaining 27 adverse events, and the final results showed that there was no significant difference in the probability of these adverse events between the zonisamide group and the control group, both for PD patients and DLB patients.

## 5. Discussion

This systematic review and meta-analysis of seven RCTs were conducted to determine the efficacy and safety of zonisamide in the treatment of PD and DLB. The UPDRS III total score was used as the primary outcome indicator to evaluate the effect of zonisamide on PD and DLB treatment. In addition, the UPDRS II total score, daily “off” time, and UPDRS Part IV, Nos. 32, 33, and 34 were also used as secondary outcome indicators to evaluate the therapeutic effect of zonisamide in PD. A total of 33 adverse event datasets were included in the final safety analysis, and we performed a subgroup analysis of the final results to further clarify the differences in the efficacy and safety of zonisamide for PD and DLB treatment.

PD and DLB, as common neurodegenerative diseases, have been a hot topic of research in recent research. In terms of PD, from a pathophysiological standpoint, depletion of the neurotransmitter dopamine in the basal ganglia causes disruption of connections to the thalamus and motor cortex, resulting in PD [31]. Dopamine replacement therapy, represented by levodopa, is the current gold standard of treatment options for PD. However, the therapeutic efficacy of dopamine begins to wear off as the disease progresses, with the emergence of “off” periods and dopamine-induced dyskinesia [32]. Given that DLB and PD share a similar pathology and that both are considered to be on the same spectrum as Lewy body disease, levodopa is also often considered for the treatment of dyskinesia in patients with DLB [33]. However, due to the nature of the disease itself, people with DLB are vulnerable to adverse effects on their own cognition and behavior and even to psychosis and psychiatric disorders, when treated with dopaminergic therapy [34, 35]. Zonisamide was approved as an antiparkinsonian drug in Japan in 2009, with its pharmacological mechanisms including dopaminergic [36, 37], nondopaminergic [38, 39], and neuroprotective effects [40], which may be associated with the improvement of PD and DLB. However, the exact mechanism of action of zonisamide in improving PD and DLB is still unclear, and more research is needed to clarify it.

The UPDRS (Unified Parkinson's Disease Rating Scale) was used to rate the clinical condition of Parkinson's disease and consists of four main components. The UPDRS Part II displays the self-assessment of patients for activities of daily life, whereas the UPDRS Part III is physician's evaluation of the patient's motor function. The UPDRS Part IV is the patient's evaluation of their own dyskinesia, with subscales 32, 33, and 34 corresponding to the duration of dyskinesia (based on nonsleep time), degree of disability caused by dyskinesia, and the degree of pain provoked by dyskinesia, respectively [41].

In this meta-analysis, our results show that treatment with zonisamide provoked an obvious decrease in both PD and DLB patients' UPDRS Part III total scores. These motor changes measured by the UPDRS Part III also confirm the significant improvement in motor function of zonisamide in PD and DLB patients. In addition, to further clarify whether the effects of zonisamide differed between PD and DLB, a subgroup analysis was performed on the final figures. Our results showed that the improvement in motor function with zonisamide was significant for both PD and DLB. And we also found that the effect of zonisamide in improving the UPDRS III total score appears to be more pronounced for DLB patients by comparing the difference. In animal studies, zonisamide was found to significantly slow the degeneration of nigral dopamine neurons caused by the expression of A53T-synuclein [42]. In a separate study, it was discovered that combining zonisamide with levodopa-carbidopa increased DOPAC levels by 300% when compared to levodopa-carbidopa treatment alone [43]. Zonisamide has also been found to delay degeneration, increase dopamine stores, and enhance dopamine release from striatal nerve endings [44], and we consider that these properties appear to explain the significant improvement in motor function of zonisamide in PD and DLB patients; however, we believe that more studies are still needed to demonstrate the superiority of zonisamide in improving motor function in DLB patients.

In addition, for PD patients, we obtained results showing that treatment with zonisamide also significantly reduced the UPDRS Part II total scores in PD patients. This shows a significant improvement in the function of daily activities in PD patients after treatment with zonisamide, which also seems to indicate that the effect of zonisamide on PD patients is not limited to motor function alone. In three other recent small open-label studies, adjunctive treatment with zonisamide also showed positive improvements in nonmotor symptoms of PD such as impulse control disorder (ICD), binge eating, and refractory anxiety [45, 46]. Therefore, after comprehensive consideration, we conclude that the ameliorative effect of zonisamide on PD is multifaceted, which also needs to be proven by more clinical studies.

For patients with PD, long-term use of levodopa can cause motor complications such as wearing off and dyskinesia. In this meta-analysis, our results showed that zonisamide treatment significantly reduced the daily “off” time, demonstrating that zonisamide could obviously improve wearing off. This may be due to the fact that zonisamide has a half-life of around 60 h, and that its plasma concentration is unaffected by dosing intervals or dosage regimen [47]. For levodopa treatment-induced dyskinesia, our findings showed a significant decrease in UPDRS Part IV, No. 32 worsened after zonisamide treatment. Furthermore, the scores for other items, including improved, no new onset, unchanged with scores ≥ 1, and new onset, to a large extent, also demonstrated improvements of zonisamide on the duration of dyskinesia, although not statistically significant. Additionally, our results showed no statistically significant difference in the effect of zonisamide use on the UPDRS Part IV, Nos. 33 and 34 compared to controls and changes. These parameters suggest that zonisamide appears to improve the duration of dyskinesia. However, its effect on pain and disability caused by dyskinesia needs to be supported by further research data and results.

In terms of safety, our final analysis showed that zonisamide was only statistically significant in terms of increasing the incidence of contusions, and by subgroup analysis, we further found that zonisamide did significantly increase the incidence of contusions in DLB, but the effect of zonisamide on contusions was not statistically significant in the subgroup analysis of PD. In addition, subgroup analysis also showed that zonisamide significantly increased the incidence of reduced appetite in DLB, and that zonisamide significantly increased the incidence of somnolence in PD. However, in the overall analysis, the effect of zonisamide on both reduced appetite and the onset of somnolence was nonsignificant. To summarize the above, in terms of safety, we consider that the use of zonisamide increases the probability of contusion in patients with DLB. In addition to a possible increase in the probability of reduced appetite in patients with DLB and somnolence in patients with PD, which need to be verified by further pilot studies, for patients with DLB, the question of whether therapeutic drugs may have adverse effects on cognitive and psychiatric symptoms is a key safety issue, and, in previous clinical studies of zonisamide in the treatment of epilepsy, it was found that zonisamide use may cause psychiatric and cognitive adverse effects [24]. Based on the above considerations, in a recent 52-week randomized controlled trial, the investigators used the NPI-10 (Neuropsychiatric Inventory) and the MMSE (Mental State Examination Scale) to measure the mental status and cognitive level of patients before and after long-term treatment with zonisamide and did not observe significant changes or deterioration in the mean NPI-10 and MMSE scores [29]. Therefore, zonisamide has a relatively reliable safety profile for the treatment of PD and DLB compared to levodopa.

The above discussion of safety is based on the effects of 25 mg and 50 mg doses of zonisamide in patients with PD and DLB. In the initial clinical study of zonisamide for PD, therapeutic amounts of 100 mg and above have also been used to try. Because the higher dose group was linked to more side effects and a nonsignificant improvement in UPDRS III scores, subsequent researchers reduced the zonisamide dose group to 25 mg and 50 mg in clinical trials [24]. The same dose setting was also used in a clinical study of zonisamide for DLB. We summarized the results of the subsequent clinical trials and discovered that both the 25 mg and 50 mg doses of zonisamide had a significant and comparable effect on motor symptoms in PD patients. However, for the wearing off in PD patients, the ameliorating effect of the 50 mg dose of zonisamide appears to be more pronounced, and PD patients appear to be more responsive to the 50 mg dose of zonisamide. The most recent study concluded that zonisamide 25 or 50 mg/day is effective in the long-term treatment of DLB patients, and that both doses are well tolerated with no new safety concerns [29]. We concluded that 25 mg and 50 mg doses of zonisamide are relatively safe and provide good improvement in the treatment of both PD and DLB, but perhaps more dose options should also be tried in future trials to explore for the highest patient benefit.

In the field of aging medicine, Parkinson's disease and dementia with Lewy bodies are currently hot topics. There are still disadvantages to levodopa therapy that need to be improved. There is currently no meta-analysis of zonisamide in the treatment of PD and DLB. As we all know, this is the first meta-analysis to assess the role of zonisamide in PD and DLB. The advantage of this analysis is that it comprehensively assesses the roles of zonisamide in activities of daily living, motor function, daily “off” time, duration of dyskinesia, disability caused by dyskinesia, and painful dyskinesia. However, our study has several limitations: (a) seven studies were all carried out on the Japanese population. Other large international multicenter clinical trials with similar reproducible findings are still lacking. (b) The follow-up periods in the included studies were brief, lasting no more than a year. There is no evidence that zonisamide treatment for more than a year results in additional histological benefits. The long-term prognosis and safety of zonisamide are still unknown, and more research is needed. (c) In three RCTs, the subjects of the studies were DLB. Enrolling patients in a long-term trial under double-blind conditions would be difficult due to the progressive nature of DLB and associated caregiver burden and could result in significant study dropouts, especially in the placebo group. (d) Since 2008, the MDS-UPDRS has been used as the new official Parkinson's Disease Rating Scale. However, the UPDRS scale, developed in 1987, was used consistently in all seven RCTs. Because the MDS-UPDRS scale may be more easily understood and answered by patients, it is also possible that differences in the content of the two scales may affect the accuracy of the final data.

## 6. Conclusions

In conclusion, we completed the current statistical analysis of outcome data on zonisamide in RCTs in PD and DLB. The combined data from RCT studies showed that zonisamide significantly improves the motor function in PD and DLB. Furthermore, in patients with PD, zonisamide has a significant positive impact on the improvement of activities of daily life, wearing off, and duration of dyskinesia. In terms of safety, the use of zonisamide significantly increases the probability of contusion in patients with DLB and may increase the probability of reduced appetite in patients with DLB and somnolence in patients with PD. In order to better guide clinical practice, more RCTs of longer duration and larger sample sizes are needed to determine the efficacy and safety of zonisamide in PD and DLB.

## Figures and Tables

**Figure 1:** PRISMA flow chart.

**Figure 2:** (a, b) Quality assessment of included studies.

**Figure 3:** The effect of zonisamide on UPDRS III total score (a), UPDRS III total score subgroup analysis (b), the effect of zonisamide on UPDRS II “Off” total score (c), the effect of zonisamide on daily “Off” time (d), and daily “Off” time subgroup analysis (e).

**Figure 4:** The effect of zonisamide on UPDRS Part IV, No. 32 worsened (a), the effect of zonisamide on UPDRS Part IV, No. 32 improved (b), the effect of zonisamide on UPDRS Part IV, No. 32 no new onset (c), the effect of zonisamide on UPDRS Part IV, No. 32 unchanged with scores ≥ 1 (d), and the effect of zonisamide on UPDRS Part IV, No. 32 new onset (e).

**Figure 5:** The effect of zonisamide on UPDRS Part IV, No. 33 worsened (a), the effect of zonisamide on UPDRS Part IV, No. 33 improved (b), the effect of zonisamide on UPDRS Part IV, No. 33 unchanged with scores ≥ 1 (c), and the effect of zonisamide on UPDRS Part IV, No. 33 zero (d).

**Figure 6:** The effect of zonisamide on UPDRS Part IV, No. 34 worsened (a), the effect of zonisamide on UPDRS Part IV, No. 34 improved (b), the effect of zonisamide on UPDRS Part IV, No. 34 unchanged with scores ≥ 1 (c), and the effect of zonisamide on UPDRS Part IV, No. 34 zero (d).

**Figure 7:** Contusion (a), contusion subgroup analysis (b), somnolence (c), and somnolence subgroup analysis (d).

**Figure 8:** Reduced appetite (a), reduced appetite subgroup analysis (b), weight loss (c), and weight loss subgroup analysis (d).

**Figure 9:** Constipation (a), constipation subgroup analysis (b), insomnia (c), and insomnia subgroup analysis (d).

## Data Availability

The article/Supplementary Material (available here) contains the original contributions presented in the study. Any additional questions should be directed to the corresponding author.

## Supplementary Materials

Supplementary Materials The supplementary materials are divided into four parts. Supplementary Material 1 is the PRISMA checklist for this meta-analysis. Supplementary Material 2 is the retrieval formula used in database search. Supplementary Material 3 describes the study's characteristics in detail. Supplementary Material 4 contains an analysis of other 27 adverse event datasets.

## References

[1] Jayaramayya K., Iyer M., Venkatesan D. (2020). Unraveling correlative roles of dopamine transporter (DAT) and Parkin in Parkinson's disease (PD) - a road to discovery. *Brain Research Bulletin*.

[2] Mohana Devi S., Mahalaxmi I., Aswathy N. P., Dhivya V., Balachandar V. (2020). Does retina play a role in Parkinson's disease?. *Acta Neurologica Belgica*.

[3] de Lau L. M., Breteler M. M. (2006). Epidemiology of Parkinson’s disease. *Lancet Neurology*.

[4] Postuma R. B., Berg D., Stern M. (2015). MDS clinical diagnostic criteria for Parkinson's disease. *Movement Disorders*.

[5] Chen R. C., Chang S. F., Su C. L. (2001). Prevalence, incidence, and mortality of PD: a door-to-door survey in Ilan County, Taiwan. *Neurology*.

[6] McKeith I., Mintzer J., Aarsland D. (2004). Dementia with Lewy bodies. *The Lancet Neurology*.

[7] Zaccai J., McCracken C., Brayne C. (2005). A systematic review of prevalence and incidence studies of dementia with Lewy bodies. *Age and Ageing*.

[8] Galasko D. (2017). Lewy Body Disorders. *Neurologic Clinics*.

[9] Gomperts S. N. (2016). Lewy body dementias: dementia with lewy bodies and parkinson disease dementia. *Continuum: Lifelong Learning in Neurology*.

[10] Tran T. N., Vo T. N. N., Frei K., Truong D. D. (2018). Levodopa-induced dyskinesia: clinical features, incidence, and risk factors. *Journal of Neural Transmission (Vienna)*.

[11] Pahwa R., Isaacson S., Jimenez-Shaheed J. (2019). Impact of dyskinesia on activities of daily living in Parkinson's disease: results from pooled phase 3 ADS-5102 clinical trials. *Parkinsonism & Related Disorders*.

[12] Coelho M., Abreu D., Correia-Guedes L. (2017). Disability in activities of daily living and severity of dyskinesias determine the handicap of Parkinson's disease patients in advanced stage selected to DBS. *Journal of Parkinson's Disease*.

[13] Pechevis M., Clarke C. E., Vieregge P. (2005). Effects of dyskinesias in Parkinson's disease on quality of life and health-related costs: a prospective European study. *European Journal of Neurology*.

[14] Vijiaratnam N., Foltynie T. (2020). Therapeutic strategies to treat or prevent off episodes in adults with Parkinson's disease. *Drugs*.

[15] McKeith I. G., Boeve B. F., Dickson D. W. (2017). Diagnosis and management of dementia with Lewy bodies: fourth consensus report of the DLB consortium. *Neurology*.

[16] Jellinger K. A., Korczyn A. D. (2018). Are dementia with Lewy bodies and Parkinson's disease dementia the same disease?. *BMC Medicine*.

[17] Reimers A., Ljung H. (2019). An evaluation of zonisamide, including its long-term efficacy, for the treatment of focal epilepsy. *Expert Opinion on Pharmacotherapy*.

[18] Li C., Xue L., Liu Y., Yang Z., Chi S., Xie A. (2020). Zonisamide for the treatment of Parkinson disease: a current update. *Frontiers in Neuroscience*.

[19] Oki M., Kaneko S., Morise S. (2017). Zonisamide ameliorates levodopa-induced dyskinesia and reduces expression of striatal genes in Parkinson model rats. *Neuroscience Research*.

[20] McElroy S. L., Kotwal R., Guerdjikova A. I. (2006). Zonisamide in the treatment of binge eating disorder with obesity: a randomized controlled trial. *The Journal of Clinical Psychiatry*.

[21] Rapoport A. M., Bigal M. E. (2004). Preventive migraine therapy: what is new. *Neurological Sciences*.

[22] Liberati A., Altman D. G., Tetzlaff J. (2009). The PRISMA statement for reporting systematic reviews and meta-analyses of studies that evaluate healthcare interventions: explanation and elaboration. *BMJ*.

[23] Tao X., Zhang Z., Yang Z., Rao B. (2022). The effects of taurine supplementation on diabetes mellitus in humans: a systematic review and meta-analysis. *Food Chemistry: Molecular Sciences*.

[24] Murata M., Hasegawa K., Kanazawa I., The Japan Zonisamide on PD Study Group (2007). Zonisamide improves motor function in Parkinson disease: a randomized, double-blind study. *Neurology*.

[25] Murata M., Hasegawa K., Kanazawa I. (2015). Zonisamide improves wearing-off in Parkinson's disease: a randomized, double-blind study. *Movement Disorders*.

[26] Murata M., Odawara T., Hasegawa K. (2018). Adjunct zonisamide to levodopa for DLB parkinsonism: a randomized double-blind phase 2 study. *Neurology*.

[27] Ikeda K., Yanagihashi M., Miura K. (2018). Zonisamide cotreatment delays striatal dopamine transporter reduction in Parkinson disease: a retrospective, observational cohort study. *Journal of the Neurological Sciences*.

[28] Murata M., Odawara T., Hasegawa K. (2020). Effect of zonisamide on parkinsonism in patients with dementia with Lewy bodies: a phase 3 randomized clinical trial. *Parkinsonism & Related Disorders*.

[29] Odawara T., Hasegawa K., Kajiwara R. (2022). Long-term efficacy and safety of zonisamide for treatment of parkinsonism in patients with dementia with Lewy bodies: an open-label extension of a phase three randomized controlled trial. *The American Journal of Geriatric Psychiatry*.

[30] Murata M., Hasegawa K., Kanazawa I. (2016). Randomized placebo‐controlled trial of zonisamide in patients with Parkinson’s disease. *Neurology and Clinical Neuroscience*.

[31] Cacabelos R. (2017). Parkinson’s disease: from pathogenesis to pharmacogenomics. *International Journal of Molecular Sciences*.

[32] Goel A., Sugumaran R., Narayan S. K. (2021). Zonisamide in Parkinson's disease: a current update. *Neurological Sciences*.

[33] Goldman J. G., Goetz C. G., Brandabur M., Sanfilippo M., Stebbins G. T. (2008). Effects of dopaminergic medications on psychosis and motor function in dementia with Lewy bodies. *Movement Disorders*.

[34] Boeve B. F., Silber M. H., Ferman T. J. (2013). Clinicopathologic correlations in 172 cases of rapid eye movement sleep behavior disorder with or without a coexisting neurologic disorder. *Sleep Medicine*.

[35] Boeve B. F., Molano J. R., Ferman T. J. (2011). Validation of the Mayo Sleep Questionnaire to screen for REM sleep behavior disorder in an aging and dementia cohort. *Sleep Medicine*.

[36] Okada M., Kaneko S., Hirano T. (1995). Effects of zonisamide on dopaminergic system. *Epilepsy Research*.

[37] Uemura M. T., Asano T., Hikawa R., Yamakado H., Takahashi R. (2017). Zonisamide inhibits monoamine oxidase and enhances motor performance and social activity. *Neuroscience Research*.

[38] Murata M. (2004). Novel therapeutic effects of the anti-convulsant, zonisamide, on Parkinson's disease. *Current Pharmaceutical Design*.

[39] Miwa H., Koh J., Kajimoto Y., Kondo T. (2011). Effects of T-type calcium channel blockers on a parkinsonian tremor model in rats. *Pharmacology, Biochemistry, and Behavior*.

[40] Terada T., Yokokura M., Yoshikawa E. (2016). Extrastriatal spreading of microglial activation in Parkinson's disease: a positron emission tomography study. *Annals of Nuclear Medicine*.

[41] Fish JJEoCN (2018). *Unified Parkinson’s disease rating scale*.

[42] Arawaka S., Fukushima S., Sato H. (2014). Zonisamide attenuates *α*-synuclein neurotoxicity by an aggregation-independent mechanism in a rat model of familial Parkinson's disease. *PLoS One*.

[43] Duty S., Jenner P. (2011). Animal models of Parkinson's disease: a source of novel treatments and clues to the cause of the disease. *British Journal of Pharmacology*.

[44] Gluck M. R., Santana L. A., Granson H., Yahr M. D. (2004). Novel dopamine releasing response of an anti-convulsant agent with possible anti-Parkinson's activity. *Journal of Neural Transmission (Vienna)*.

[45] Bermejo P. E., Ruiz-Huete C., Anciones B. (2010). Zonisamide in managing impulse control disorders in Parkinson's disease. *Journal of Neurology*.

[46] Kinrys G., Vasconcelos e Sa D., Nery F. (2007). Adjunctive zonisamide for treatment refractory anxiety. *International Journal of Clinical Practice*.

[47] D'Amico D. (2007). Antiepileptic drugs in the prophylaxis of migraine, chronic headache forms and cluster headache: a review of their efficacy and tolerability. *Neurological Sciences*.

